The article "Homocysteinylated Albumin Promotes Increased Monocyte-Endothelial Cell Adhesion and Up-Regulation of MCP1, Hsp60 and ADAM17" was retracted in 2019. Reason: duplicate publication.

# Homocysteinylated Albumin Promotes Increased Monocyte-Endothelial Cell Adhesion and Up-Regulation of MCP1, Hsp60 and ADAM17

**DOI:** 10.1371/journal.pone.0031388

**Published:** 2012-02-03

**Authors:** Rosanna Capasso, Irene Sambri, Amelia Cimmino, Sofia Salemme, Cinzia Lombardi, Filomena Acanfora, Ersilia Satta, Donald L. Puppione, Alessandra F. Perna, Diego Ingrosso

**Affiliations:** 1 Department of Biochemistry and Biophysics “F. Cedrangolo”, School of Medicine, Second University of Naples, Naples, Italy; 2 Cardiovascular Research Centre, School of Medicine, Second University of Naples, Naples, Italy; 3 First Division of Nephrology, School of Medicine, Second University of Naples, Naples, Italy; 4 Institute of Genetics and Biophysics, National Research Council, Naples, Italy; 5 The Molecular Biology Institute, University of California Los Angeles, Los Angeles, California, United States of America; Idaho State University, United States of America

## Abstract

**Rationale:**

The cardiovascular risk factor homocysteine is mainly bound to proteins in human plasma, and it has been hypothesized that homocysteinylated proteins are important mediators of the toxic effects of hyperhomocysteinemia. It has been recently demonstrated that homocysteinylated proteins are elevated in hemodialysis patients, a high cardiovascular risk population, and that homocysteinylated albumin shows altered properties.

**Objective:**

Aim of this work was to investigate the effects of homocysteinylated albumin - the circulating form of this amino acid, utilized at the concentration present in uremia - on monocyte adhesion to a human endothelial cell culture monolayer and the relevant molecular changes induced at both cell levels.

**Methods and Results:**

Treated endothelial cells showed a significant increase in monocyte adhesion. Endothelial cells showed after treatment a significant, specific and time-dependent increase in ICAM1 and VCAM1. Expression profiling and real time PCR, as well as protein analysis, showed an increase in the expression of genes encoding for chemokines/cytokines regulating the adhesion process and mediators of vascular remodeling (ADAM17, MCP1, and Hsp60). The mature form of ADAM17 was also increased as well as Tnf-α released in the cell medium. At monocyte level, treatment induced up-regulation of ICAM1, MCP1 and its receptor CCR2.

**Conclusions:**

Treatment with homocysteinylated albumin specifically increases monocyte adhesion to endothelial cells through up-regulation of effectors involved in vascular remodeling.

## Introduction

Hyperhomocysteinemia is a cardiovascular risk factor both in the general population and in selected patient groups [1]. Previous evidence showed that high homocysteine increases cell adhesion and induces a proinflammatory state in the vessel wall by promoting adhesion molecule expression and monocyte recruitment. In particular, nuclear factor (NF)-kB activation and intercellular adhesion molecule-1 (ICAM-1) stimulation have been shown [2]. High homocysteine also up-regulates monocyte chemoattractant protein-1 (MCP1), interleukin-8 (IL-8) expression and secretion in cultured human endothelial cells, smooth muscles cells, and monocytes [3]–[6]. Also VCAM-1 expression is up-regulated [7].

The article "Homocysteinylated Albumin Promotes Increased Monocyte-Endothelial Cell Adhesion and Up-Regulation of MCP1, Hsp60 and ADAM17" was retracted in 2019. Reason: duplicate publication.

Plasma homocysteine is mainly protein-bound, accounting for >90% of total homocysteine (the remainder is found as free low-molecular weight disulfide forms, including homocystine, that is the homocysteine homodimer, and the homocysteine-cysteine mixed disulfide). Only 1.5–4% of homocysteine in circulation is present in its reduced form [8]. In many of previous studies, homocysteine was simply added to cell culture medium in its rather unphysiological free reduced form, thus rising concerns about the possibility of artifactual effects mediated through intervening formation of adducts with unpredictable protein targets.

Under physiological conditions protein homocysteinylation occurs through acylation of free amino groups (protein-*N*-homocysteinylation), [9]–[11] and thiol group oxidation (protein-*S*-homocysteinylation) [12].

It has been shown that hyperhomocysteinemia elicits its effects on the vasculature mainly through homocysteinylated proteins [13]. In this respect, the functional properties of human serum albumin are altered by homocysteine binding [14].

Homocysteine is commonly elevated in end-stage renal disease (ESRD) patients on hemodialysis. This fact has attracted much scientific interest, because of the high cardiovascular risk in these patients, which is not exhaustively explained by the presence of conventional risk factors and/or specific uremic toxins [15]–[17]. We recently showed that plasma protein homocysteinylation is increased in uremic patients on hemodialysis and significantly reduced, although not normalized, after folate supplementation [14]. Concerning this issue, it can be mentioned that some emphasis has been given in the literature on the role played by protein-bound uremic toxins [18].

Protein homocysteinylation could be one of the principal mediators of homocysteine toxicity, contributing to detrimental structural and functional alterations at the molecular and cellular level [19]–[21]. We therefore investigated the role of homocysteinylated albumin in eliciting cell adhesion, and monitored, starting with a genome-wide approach, the expression of relevant mediators in the adhesion process.

The article "Homocysteinylated Albumin Promotes Increased Monocyte-Endothelial Cell Adhesion and Up-Regulation of MCP1, Hsp60 and ADAM17" was retracted in 2019. Reason: duplicate publication.

## Methods

### Synthesis and characterization of homocysteinylated albumin

Homocysteinylated albumin was produced according to a modification of the protocol published by Jakubowski [9] by incubation with homocysteine thiolactone, determining the formation of mainly *N*-homocysteinylated albumin, and a smaller amount of *S*-homocysteinylated albumin. Homocysteinylated albumin was HPLC-analyzed [14]. The *N*-homocysteinylated albumin adduct was largely prevalent, while a very small amount of *S*-homocysteinylated albumin. *N*-homocysteinylated albumin concentrations used in the experiments were in the range of 0.80 nmol Hcy/mg albumin and, in order to facilitate comparison with equivalent concentrations of circulating *N*-protein bound homocysteine, are referred to as equivalent to concentration of homocysteine in mol/L [14].

Homocysteinylated and unmodified albumin, purified by reversed phase HPLC [14], were then characterized by electrospray mass spectrometry (ESI-MS) at the Pasarow Mass Spectrometry Laboratory, UCLA, Los Angeles California, U.S.A., as described by Puppione et al. [22]. Briefly, samples were separated by size-exclusion chromatography and mass spectrometry (ESI-MS) was performed using a triple quadrupole instrument (API III, Applied Biosystems). Data were processed using MacSpec 3.3, Hypermass and BioMultiview 1.3.1 software (Applied Biosistems).

### Cell cultures and treatments

Human endothelial cell line EAhy926 (ATCC) were grown in high glucose concentration DMEM (Gibco), containing 10% fetal bovine serum (Gibco), 1% glutamine, 1% penicillin/streptomycin (Gibco), 1% fungizone (Gibco). Human monocytoid cell line U937 (ATCC) were grown in RPMI-1640 (Gibco) containing 10% bovine fetal serum (Gibco), 1% penicillin/streptomycin (Gibco).

EAhy926 were incubated for 18 h, in the presence of 0.3 or 1.0 µmol/L Homocysteinylated albumin equivalent. Negative controls were: a) cells incubated with unmodified human serum albumin at a comparable protein concentration; b) cells incubated without human serum albumin (*i.e.* untreated negative control); c) cells incubated with carboxylmethylated human serum albumin, as a control of differently-modified albumin at cysteine levels [23]. This control was included in order to rule out that any covalent modification of human serum albumin could trigger adhesion, irrespective of the kind of amino acid modification involved. Cells incubated with Tnf-α 10 ng/ml for 4 h represented positive controls.

U937 (ATCC) were incubated for 18 h, in the presence of 1.0 µmol/L Homocysteinylated albumin equivalent. Negative controls were: a) cells incubated with unmodified human serum albumin at a comparable protein concentration; b) cells incubated without human serum albumin (*i.e.* untreated negative control).

The article "Homocysteinylated Albumin Promotes Increased Monocyte-Endothelial Cell Adhesion and Up-Regulation of MCP1, Hsp60 and ADAM17" was retracted in 2019. Reason: duplicate publication.

### Adhesion assay

EAhy926 were plated to 90% confluence in 24-well multiwell plates and treated with homocysteinylated albumin or the appropriate control for 18 h at 37°C. Treatment medium was removed and saved; cells were washed once with incomplete DMEM medium and 8×10^5^ monocytoid cells per well were co-incubated, for 30 min at 37°C in the endothelial treatment medium. Non-adherent U937 were removed by gently washing thrice with PBS. Finally PBS containing 1% glutaraldehyde was added to fix monocytes to the endothelial monolayer. Adherent monocytes were counted directly using a Zeiss Axiovert 10 inverted photomicroscope (Carl Zeiss S.p.A., Milan, Italy) on three randomly selected high magnification microscopic fields per well, for each independent experiment. Ten independent experiments were performed. Results were expressed as both mean of the absolute number of adherent monocytes per field, and percentage of adherent monocytes relevant to samples treated with Tnf-α (100% adhesion).

### RNA extraction

RNA extraction was performed, on endothelial cells, treated with homocysteinylated albumin, utilizing Trizol reagent (Invitrogen), according to the supplier's protocols. RNA concentration was measured by NanoDrop UV/VIS micro- spectrophotometry (ND-*1000*; NanoDrop Technologies, Wilmington, DE, USA).

### Expression profile

Microrray hybridization and data analysis were carried out using Human Genome U133A Plus 2.0 GeneChip arrays (Affymetrix, Santa Clara, CA, U.S.A.), containing 54000 hybridized genes, essentially as described by Calin et al [24]. Transcriptome data were compliant with the MIAME (Minimum Information About a Microarray Experiment) standard and registered in suitable format on the ArrayExpress Archive database (http://www.ebi.ac.uk/microarray-as/ae/).

### Real time PCR

cDNA synthesis from 1 µg of total RNA was made using the QuantiTect reverse transcriptase kit (Qiagen, Life Sciences, Milan, Italy). Amplifications were performed with the iCycler thermalcycler (Bio-Rad Laboratories S.r.l., Segrate Milan, Italy) with the fluorescence detection system iCycler iQ real time PCR. The amplification mix contained 1 µl cDNA, 0.3 µM of each primer, 12.5 µl of master mix QuantiTECT SYBR green (Quiagen), and H_2_O DEPC, for a final volume of 25 µl. Primers pair and amplification condition are described in Table 1. Relative expression was calculated using the delta Cq method. The value of 2^−delta delta Cq^>1 reflects increased expression of the relevant gene, and a value of 2^−delta delta Cq^<1 points to a decrease in gene expression.

The article "Homocysteinylated Albumin Promotes Increased Monocyte-Endothelial Cell Adhesion and Up-Regulation of MCP1, Hsp60 and ADAM17" was retracted in 2019. Reason: duplicate publication.

**Table 1:** Amplification conditions and primer pairs for PCR experiments.

***MCP1*** (NM_002982.3)	95°C for 30 sec, 58°C for 30 sec, 72°C for 30 sec
	5′-CAGCAGCAAGTGTCCCAAAG-3′
	5′-GAGTGAGTGTTCAAGTCTTCGG-3′
***ICAM1*** (NM_000201)	95°C for 30 sec, 62°C for 30 sec, 72°C for 30 sec
	5′-GGTGTATGAACTGAGCAATGTG-3′
	5′-TGGCAGCGTAGGGTAAGG-3′
***ADAM17*** (NM_003183)	95°C for 30 sec, 55°C for 30 sec, 72°C for 30 sec
	5′-GTATCTGAACAACGACACCTG-3′
	5′-CTCCTGGCACTTCTTCTGG-3′
***NRP1*** (NM_003873)	95°C for 30 sec, 60°C for 30 sec, 72°C for 30 sec
	5′-GGAACTTGGTGGATGAATGTGATG-3′
	5′-CTCTGATTGTATGGTGCTGTCTATG-3′
***TFP1*** (NM_006287)	95°C for 30 sec, 57°C for 30 sec, 72°C for 30 sec
	5′-ATAACTCCCTGACTCCGCAATC-3′
	5′-TGGCACGACACAATCCTCTG-3′
***VCAM1*** (NM_001078)	95°C for 30 sec, 63°C for 30 sec, 72°C for 30 sec
	5′-TCTACGCTGACAATGAATCCTG-3′
	5′-CTTGACTGTGATCGGCTTCC-3′
***CCR2*** (NM_001123396)	95°C for 30 sec, 54°C for 30 sec, 72°C for 30 sec
	5′-TTCTTCATCATACTCCTGACAATCG-3′
	5′-AGCAAACACAGCCACCAACC-3′
***Hsp60***	95°C for 30 sec, 55°C for 30 sec, 72°C for 30 sec
	Quatitect primer assay (Quiagen)

All conditions are relevant to real time PCR except for *VCAM1*, where tradition PCR has been employed. 35 amplification cycles have been performed.

For VCAM1 transcript amplification, 2 µl cDNA were employed and mix was replaced by a mixture containing: 0.5unit of Taq Polymerase (Fermentas Inc., MD, USA), 0.2 mM each dNTP, 2 µl buffer, in a 20 µl final volume and reactions carried out in a Mastercycler gradient (Eppendorf s.r.l., Milan, Italy).

### Protein analyses

Western Blot analyses were performed as previously described [25], using anti-human HSP60 (BD Pharmingen), anti-human ADAM17 (Abcam), anti-human MCP1 (Santa Cruz), anti-human ICAM1 (BD Pharmingen) and anti-human CCR2 (Abcam) as appropriate.

ICAM1, VCAM1, MCP1 and Tnf-alpha concentrations in cell culture media were determined utilizing the relevant ELISA kits (R&D Systems) according to the supplier's protocols.

Immunoprecipitation of Hsp60 was performed by magnetic bead separation using DYNAL Beads (Invitrogen) crosslinked to anti-human Hsp60 antibody (ABCAM) according to the manufacturer. The protein eluted from the crosslinked beads was revealed by Western blotting.

### Cytofluorometric analysis

Cell pellets, harvested and washed with cold PBS containing 0.1% BSA were treated with Phycoeritrine-labeled anti-VCAM1 antibodies or Allophycocyanin-labeled anti-ICAM1 (BD Pharmingen, Milan, Italy) and incubated in ice for 1 h in the dark. At the end of incubation, 1 ml of cold PBS/0.1% BSA was added and cells were pelleted. Finally, 500 µl of a PBS/0.1% BSA containing 1 µl of 0.2 µg/ml propidium iodide (Sigma-Aldrich, Milan, Italy) were added to the cell pellets prior to analysis. cytofluorimetric analysis was performed in a FACSCalibur (BD Biosciences, Milan, Italy).

The article "Homocysteinylated Albumin Promotes Increased Monocyte-Endothelial Cell Adhesion and Up-Regulation of MCP1, Hsp60 and ADAM17" was retracted in 2019. Reason: duplicate publication.

### Statistical analysis

An unpaired Student's t test was performed, to compare means in the homocysteinylated albumin experiments, or a two-way ANOVA to assess the timed effects of treatments as appropriate [26]. All results are presented as the mean (SD). All experiments were done in triplicate except otherwise stated.

## Results

### Characterization of homocysteinylated albumin by mass spectrometry

ESI-MS spectra of unmodified albumin and its homocysteinylated derivative are reported in Fig. 1. The calculated molecular mass value of native albumin was 66446 Da (Fig. 1; panel A). The homocysteinylated derivative had a calculated molecular mass of 67805 Da (Fig. 1 panel B, inset) and a calculated mass of 33903 Da for the doubly charged protein (Fig. 1; panel B). The difference between the homocysteinylated and native species is equal to 1359 Da. This difference corresponds to the acquisition of 7 *N*-homocysteinyl moieties (*N*-Lys-Hcy-*SH*; 117 Da), which are *N*-linked (amide linkage) to as many Lys residues of albumin [27], plus 4 *S*-homocysteinyl moieties (*N*-Lys-Hcy-*S*-*S*-Hcy; 133 Da), linked to *N*-linked homocysteine, through an *S-S* linkage [11], [28]–[30]. This result is highly consistent with what previously reported [27] except that the *S*-linked species could not be detected in this report, since the thiol groups in the *N*-homocysteinylated protein derivative were blocked by iodoacetamide (we omitted this step in order to prevent possible non-physiological toxic effects to cell cultures). On the other hand the reactivity of the free thiol group of the *N*-linked homocysteinyl moiety has been amply established by previous work [11], [28]–[30].

**Figure 1:** Characterization of homocysteinylated albumin by mass spectrometry. Panel A: ESI-MS of human serum albumin. Panel B: ESI-MS of homocysteinylated albumin. Inset: magnification on expanded scale of the signal at Da = 67805. The family of molecular ions is compatible with the structures shown in the panel.

### Effects of treatment of EAhy926 monolayer with homocysteinylated albumin on monocyte adhesion

Results are presented both as the mean of adherent monocyte number per field (Fig. 2A), and as percent of adhesion with respect to the Tnf-α treated positive control (100% adhesion) (Fig. 2B). Examples of adhesion assay presentation are also given (Fig. 2C).

**Figure 2:** Effects of homocysteinylated albumin on monocyte adhesion. U937 monocytoid cells adhesion onto an endothelial monolayer (EAhy926) expressed as adherent cells (number/field; panel A) and percentage adherent cells compared to positive control (panel B). Counts are the mean of ten independent experiments, each carried out by counting five different fields/sample of triplicate samples. Examples of microscopic fields are shown on the right. C: negative control (untreated cells); A: unmodified albumin; AH: homocysteinylated albumin; AC: carboxymethylated albumin; T: positive control (Tnf-α). 0.3 or 1: homocysteine micromolar concentration present in the assay in the form of *N*-homocysteinyl groups bound to albumin, as comparable to the in vivo situation [14]; p<0.0001.

The article "Homocysteinylated Albumin Promotes Increased Monocyte-Endothelial Cell Adhesion and Up-Regulation of MCP1, Hsp60 and ADAM17" was retracted in 2019. Reason: duplicate publication.

Results showed that treatment of endothelial cells with Homocysteinylated albumin at concentrations comparable to those detected *in vivo* in uremic hyperhomocysteinemic patients [14] is followed by a significant increase of monocyte adhesion onto the endothelial monolayers. Conversely, treatment with Homocysteinylated albumin, at concentrations comparable to those detected *in vivo* [14] in normal subjects, does not result in any significant increase of adhesion with respect to control treatments.

### Homocysteinylated albumin treatment increases adhesion molecule expression

Cell adhesion and endothelial damage are increased in uremia and paralleled by time-dependent VCAM-1 and ICAM-1 up-regulation [31], [32].

Fig. 3 and 4 show the results of ICAM1 and VCAM1 kinetic monitoring in Eahy926 treated with 1.0 µmol/L homocysteinylated albumin compared to control at both gene expression and protein levels. *ICAM1* transcripts significantly increased after 1.0 µmol/L homocysteinylated albumin treatment, compared to control (Fig. 3A). Consistently, a significant increase in the surface expression of ICAM1 protein became evident within 18 h treatment (Fig. 3B), paralleled by ICAM1 release in the medium (Fig. 3C), thus mirroring the situation detected at cell surface level.

**Figure 3:** ICAM1 expression in endothelial cells treated with N-homocysteinylated albumin. Panel A: expression levels of ICAM1 transcripts quantitated by real time PCR (treated: 1 µmol/L homocysteinylated albumin; control: unmodified albumin); (p<0.001). Panel B: cytofluorimetric analysis of ICAM1 time course surface expression by EAhy926 endothelial cells treated with homocysteinylated albumin (C: unmodified albumin negative control; Tnf-α: positive control). Panel C: Time course of ICAM1 release in the culture medium, quantitated by ELISA assay. C: negative control (untreated cells); A: unmodified albumin; AH: 1 µmol/L homocysteinylated albumin; (p<0.001).

**Figure 4:** VCAM1 expression in endothelial cells treated with N-homocysteinylated albumin. Panel A: Time course of induction of VCAM1 transcripts, in EAhy926 endothelial cells, by treatment with 1 µmol/L homocysteinylated albumin. Panel B: cytofluorimetric analysis of ICAM1 time course surface expression by EAhy926 endothelial cells treated with homocysteinylated albumin. (C: unmodified albumin negative control; Tnf-α: positive control). Panel C: Time course of ICAM1 release in the culture medium, quantitated by ELISA assay. C: negative control (untreated cells); A: unmodified albumin; AH: 1 µmol/L homocysteinylated albumin. (p<0.001).

The article "Homocysteinylated Albumin Promotes Increased Monocyte-Endothelial Cell Adhesion and Up-Regulation of MCP1, Hsp60 and ADAM17" was retracted in 2019. Reason: duplicate publication.

After only 2 h of treatment, as shown in Fig. 4A, the *VCAM1* transcripts could be detected, and decline thereafter. This indicates that homocysteinylated albumin elicits an immediate response in the regulation of this particular gene. Also VCAM1 antigen exposure could be detected at high levels on cell surface at 18 h of treatment with homocysteinylated albumin (Fig. 4B). Consistently, a parallel increase in VCAM1 protein released in the medium could be also detected in the culture medium of cells treated with homocysteinylated albumin, compared to control (Fig. 4C).

#### Homocysteinylated albumin treatment determines increased expression in specific mediators of endothelial cell activation and damage

We were then prompted to investigate the alterations induced by homocysteinylated albumin on endothelial monolayers, which may explain the increased tendency of monocytoid cells to adhere. To this purpose we employed a genome-wide transcriptional analysis using microarray hybridization. RNA samples, extracted from endothelial cells treated with 1 µmol/L homocysteinylated albumin, untreated albumin, and untreated cells, were utilized. Treatment with homocysteinylated albumin significantly modifies gene expression profile of endothelial cells compared to control. In particular, among the twenty-three up-regulated genes, five are possibly implicated in endothelial activation (CCL2, HSPD1, ADAM17, TFP1, NRP1) (Table 2). Validation by real time PCR was carried out for MCP1, HSPD1, ADAM17, TFP1, NRP1, in consideration of their possible involvement in vascular remodeling processes. The increase of transcript levels, upon treatment with 1 µmol/L homocysteinylated albumin, was confirmed for all these five genes of interest (Fig. 5).

**Figure 5:** Validation by Q-PCR of transcriptome results relevant to upregulated gene involved in endothelial dysfunction. A: unmodified albumin; AH: homocysteinylated albumin. Gene expression in the AH sample group was significantly increased with respect to the corresponding genes in the A sample group (p<0.001).

**Table 2:** Upregulated genes from transcriptional analysis of EAhy926 cells treated with homocysteinylated albumin compared to control.

GENE NAME AND FUNCTION	GENE SYMBOL	Accession number	Fold change
Tissue Factor Pathway Inhibitor isoform a	TFP1	215447_at	4.972
NADH Dehydrogenase subunit 5	MTND5	1553575_at	4.762
Dehydrogenase/Reductase member 2 isoform 2	DHRS2	214079_at	4.711
Neuropilin1	NRP1	234072_at	4.178
Spectrin Repeat Containing Nuclear Envelop 1	SYNE1	244144_at	3.758
Insulin-like growth factor 1 receptor	IGF1R	203628_at	3.598
Secretogranin V, Variant 1	SCG5	203889_at	3.441
Xenotropic/Polytropic Retrovirus Receptor, var 1	XPR1	244755_at	3.331
Transmembr. coiled-coin domain family 1, var 3	TMCC1	237943_at	2.788
ADAM17 metalloprotease	ADAM17	205745_x_at	2.664
Tau Tubulin Kinase 2	TTBK2	231610_at	2.664
Mitochondrial Ribosomal Protein S28	MRPS28	236955_at	2.609
Dehydrogenase/Reductase member 2, var 3	DHRS2	206463_s_at	2.581
Solute Carrier Family 25, member 45, var 1	SLC25A45	1563498_s_at	2.497
RAS p21 protein activator 2	RASA2	206636_at	2.474
Polypyrimidine tract binding protein 2	PTBP2	236962_at	2.446
par-3 partitioning defective 3 homolog B, var B	PARD3B	244586_x_at	2.387
mucin20, cell surface associated, var S	MUC20	226622_at	2.374
UDP-glucose ceramide glucosyltransferase	UCGC	204881_s_at	2.265
PAP associated domain, var 1	MTPAP	238706_at	2.241
Chemokine (C-C motif) ligand 2	CCL2	216598_s_at	2.236
ubinuclein 2	UBN2	238350_at	2.140
Heat shock protein 60 kD	HSPD1	200806_s_at	2.005

Homocysteinylated albumin concentration was comparable to that detected *in vivo* in hyperhomocysteinemic uremic patients compared to control.

The article "Homocysteinylated Albumin Promotes Increased Monocyte-Endothelial Cell Adhesion and Up-Regulation of MCP1, Hsp60 and ADAM17" was retracted in 2019. Reason: duplicate publication.

Among the up-regulated genes identified in the transcriptional profile of endothelial cells treated with 1.0 µmol/L homocysteinylated albumin, we identified three genes deserving special notice for their involvement in vascular activation and damage: *CCL2*, *ADAM17*, and *Hsp60*. Transcriptional increase of all these genes (real time PCR), as well as the levels of the relevant protein products (ELISA and/or western blot), were also kinetically monitored.

A time-dependent increase in *MCP1* transcription levels could be observed, in Eahy926 treated with 1.0 µmol/L homocysteinylated albumin with a maximum at 18 h (Fig. 6A). Consistently, ELISA assays showed a significant increase in MCP1 secreted by treated cells (Fig. 6B).

**Figure 6:** Time-dependent, increased expression of ADAM17, MCP1 and Hsp60 in endothelial cells upon homocysteinylated albumin treatment. Panel A: Real time PCR evaluation during time course of *ADAM17*, *MCP1* and *Hsp60* mRNA. Panel B: ELISA assay of MCP1 released in the culture medium of treated cells. Panel C: Western blotting analysis of intracellular levels of ADAM17, and Hsp60, and analysis of Hsp60 released in the medium by immunoprecipitation and western blotting (Hsp60 IP). A: unmodified albumin control; AH: homocysteinylated albumin treatment. Levels of transcripts or proteins in the homocysteinylated albumin sample group were significantly increased compared to control (p<0.001).

The article "Homocysteinylated Albumin Promotes Increased Monocyte-Endothelial Cell Adhesion and Up-Regulation of MCP1, Hsp60 and ADAM17" was retracted in 2019. Reason: duplicate publication.

The transcript of ADAM17 is subject to time-dependent increase upon treatment of endothelial cells with 1.0 µmol/L homocysteinylated albumin (Fig. 6A). In addition, protein levels were analyzed using an antibody capable of recognizing the two forms, the precursor (110 kDa) and the mature form (80 kDa), of ADAM17 and, as shows in Fig. 6C, an increase of both ADAM17 forms could be observed, which was particularly evident in the case of the mature form. Consistently, we also found a release of Tnf-alpha in the culture medium of cells treated with homocysteinylated albumin, (168 pg/ml), while it was undetectable in the controls.

Hsp60 transcription levels also increased, in a time-dependent fashion, with a similar peak at 18 h (Fig. 6A). In consideration of the prevalent intracellular localization of Hsp60 antigen, we evaluated Hsp60 with Western blotting on endothelial cell extracts. Hsp60 is normally segregated within the intracellular compartment. We showed, by immunoprecipitation, that, upon stimulation with homocysteinylated albumin, Hsp60 increased within the intracellular compartment, paralleled by a time-dependent release of Hsp60 in the medium (Fig. 6C).

### Homocysteinylated albumin treatment determines increased expression in specific mediators on U937

Cell adhesion involves changes which occur both at the endothelial and monocyte levels. We were then prompted to investigate the alterations induced by homocysteinylated albumin on monocyte U937 cell line, under conditions in which we observed an increased cell adhesion to endothelial monolayers treated with homocysteinylated albumin. We then analyzed the expression levels and the relevant protein levels of three important markers of monocyte activation, ICAM1, MCP1 and CCR2. U937 treated with homocysteinylated albumin 1.0 µmol/L showed a significant increase both of mRNA levels (Fig. 7A) and protein levels (Fig. 7B) of ICAM1, MCP1 and CCR2, thus confirming that the observed increase in monocyte adhesion, upon treatment with homocysteinylated albumin, occurs through up-regulation of some typical mediator molecules of monocyte activation.

**Figure 7:** Increased expression of ICAM1, MCP1 and CCR2 in U937 upon homocysteinylated albumin treatment. Panel A: Real time PCR evaluation of *ICAM1*, *CCR2* and *MCP1* mRNA. Panel B: Western blotting analysis of intracellular levels of ICAM1, CCR2 and MCP1. Levels of both transcripts and proteins in the homocysteinylated albumin sample were significantly increased compared to control (p<0.001).

The article "Homocysteinylated Albumin Promotes Increased Monocyte-Endothelial Cell Adhesion and Up-Regulation of MCP1, Hsp60 and ADAM17" was retracted in 2019. Reason: duplicate publication.

## Discussion

We investigated the effects of homocysteinylated albumin treatment on monocyte adhesion in a human endothelial cell co-culture system and relevant biomolecular alterations. We observed increased monocyte adhesion onto the endothelial monolayers, concomitantly with up-regulation of ICAM-1 and VCAM-1 after treatment with homocysteinylated proteins. It has been previously shown that high homocysteine modifies gene expression in cultured cells [33]–[35] and *in vivo* in animal models [36] and in humans [37]. In our present model, both endothelial and monocytoid cells showed, after treatment, a significant, specific and time-dependent increase, at both transcriptional and protein levels, of genes potentially involved in vascular remodeling processes: *i.e.* ADAM17, MCP1, Hsp60 as schematically summarized in Fig. 8.

**Figure 8:** Summary of the effects of homocysteinylated albumin at cellular levels. Concentrations of *N*-homocysteinylated albumin, comparable to those detected *in vivo* [14], were used. Right panel: untreated cells. Left panel: treated cells. Numbers in circle refer to molecular markers and mediators of increased adhesion detected in the present work. At endothelial cell level. Transcriptional activation of MCP1, Hsp60, ADAM17 (no 1). Increase of the cleaved form of ADAM17 (no 2). Increased shedding of Tnfα (no 3), ICAM1 and VCAM1 (AM: adhesion molecules; no 4). Increased intracellular levels and release of Hsp60 (no 5). Increased MCP1 levels and release (no 6). At monocyte level. Transcriptional activation of MCP1, CCR2 and ICAM1 (no 7). Increased levels of MCP1 (no 8), CCR2 (no 9), ICAM1 (no 10). The prevalent molecular circulating homocysteine-protein adducts are schematically illustrated in the lower left corner of right panel (see also Fig. 1).

ADAM17 is a metalloproteinase involved in the shedding of adhesion molecules, *e.g.* ICAM1 [38] and Tnf-α release [39]. Transcriptional up-regulation of ADAM 17 was accompanied by an increase of its mature form, and, consistently, of Tnf-α released in the cell medium. ADAM17 activation is also consistent with the increase of ICAM1 released in the medium of treated cells. Hyperhomocysteinemia has been hypothesized to be an indicator of oxidant stress [40]. Moreover homocysteinylated, oxidized LDL-dependent increase of reactive oxygen species in the endothelium has been shown [41]. Consistently, we may hypothesize that, in our model of hyperhomocysteinemia, high homocysteinylated albumin may contribute to activation of ADAM17 through the chemical displacement of the pro-domain in the cysteine switch of this protein [42].

The article "Homocysteinylated Albumin Promotes Increased Monocyte-Endothelial Cell Adhesion and Up-Regulation of MCP1, Hsp60 and ADAM17" was retracted in 2019. Reason: duplicate publication.

We also detected an up-regulation of MCP1, a protein belonging to type CC chemokine family, that mediates monocyte recruitment in proximity of endothelial lesions, by creating of a chemotactic gradient towards the inflammatory site. Consistently, we found a significant increase of MCP1 in the medium of treated cell, compared to controls.

Homocysteinylated albumin treatment also determined a transcriptional up-regulation of Hsp60, together with its protein product. Hsp60 was increased both at the cellular level and in the extracellular medium. Heat shock proteins regulate maintenance of protein conformation and stability, through their reciprocal interaction. They can be expressed constitutively or produced in response to various types of cell stress. Hsp60 was shown to be an important autoantigen in atherosclerosis [43]. Hsp60 overexpression entails its expression on cell surface and its secretion, favoring macrophage adhesion and trans-endothelial migration. Such studies also showed that Hsp60 membrane exposure participates in the pathogenesis of the endothelial lesions by binding to specific antibodies, thus eliciting a cytotoxic effect towards the endothelium. Macrophages express Hsp60 ligands and their interaction induces their activation [44]. Plasma levels of Hsp60 are significantly higher in subjects with cardiovascular disease with respect to those without [45].

The alterations we detected in the endothelial cells, in response to homocysteinylated albumin treatment, were mirrored by consistent alterations induced in the monocytoid cells. In these cell components we detected, upon homocysteinylated albumin treatment, an up-regulation of ICAM1 and MCP1 (which are known to be produced by activated monocyte to amplify inflammatory signal reinforcing monocyte recruitment) and CCR2 (the MCP1 receptor). We previously showed that, in mononuclear cells of uremic patients on hemodialysis, who are typically hyperhomocysteinemic, DNA hypomethylation is present, with alterations of the expression pattern of methylation-dependent genes [37].

It has been previously shown that homocysteine is capable of inducing vascular alterations at endothelial and vascular smooth muscle cell levels. Hyperhomocysteinemia and hypomethylation are associated with the activation of growth factors, lipid deposition, and vascular smooth muscle cell proliferation activation. High homocysteine triggers a pro-inflammatory state involving adhesion molecule expression and monocyte recruitment, through NF-kB activation and stimulation of ICAM-1 and VCAM-1 induction [46], [47]. Homocysteine induces *in vitro*, in endothelial and vascular smooth muscle cells, increased expression of MCP1, of interleukin-8 (IL-8) and their secretion, thus promoting monocyte adhesion [2]–[7], [48]–[51]. It has been reported that hyperhomocysteinemia due to CBS deficiency promotes monocyte activation and proinflammatory alterations in transgenic mice [52]. However, previous work was often performed utilizing concentrations of free homocysteine in the high micromolar or even millimolar range, *i.e.* up to one order of magnitude higher than what observed in homocystinuria, the pathological condition in which the highest levels are reached [2]–[7], [48]–[53]. In our present work, for the first time, we treated cells with high homocysteine mimicking conditions which actually take place in vivo. In fact we carried out cell treatment with homocysteinylated albumin (not free homocysteine) and its concentrations were comparable to the *in vivo* uremic milieu.

The article "Homocysteinylated Albumin Promotes Increased Monocyte-Endothelial Cell Adhesion and Up-Regulation of MCP1, Hsp60 and ADAM17" was retracted in 2019. Reason: duplicate publication.

Homocysteine is mainly protein-bound and homocysteinylation is a widespread post-biosynthetic protein modification regarded as a major mechanism through which homocysteine induces vascular alterations. In this respect it has been shown that *N*-homocysteinylated derivatives of both LDL [21] and HDL [54] are detectable in human plasma, suggesting that homocysteinylation of plasma lipoproteins occurring *in vivo* is facilitated by lipoproteins oxidation, since these oxidized lipoprotein are more susceptible to homocysteinylation with respect to unmodified lipoproteins. It has been proposed that protein homocysteinylation could be one of the principal mediators of homocysteine toxicity [19]–[21]. We showed increased plasma protein homocysteinylation in hyperhomocysteinemic uremic patients on hemodialysis, which resulted only partially responsive to homocysteine-lowering therapy [14]. Albumin also mediates protein endocytosis, and is itself internalized, thus determining, under pathological conditions, an alteration of the expression of cytokines and relevant receptors [55], [56]. Human serum albumin displays altered functional properties (e.g. towards ligand binding) in consequence of homocysteinylation [14].

All in all our present data support the hypothesis that homocysteinylated proteins are neither secondary byproducts nor a mere biohumoral circulating marker of chronic hyperhomocysteinemia. Our data speak in favor of a mechanistic model of action according to which protein homocysteinylation, rather than free homocysteine, could exerts cell responses related to up-regulation of inflammatory chemokines which have been directly related to the pathogenesis of the early steps of atherosclerotic lesions.
